The article "Recurrent Giant Cell Tumour of Distal End Radius: Treatment and Outcomes After Further Surgeries" was published in 2022. Journal: Cureus.

# Recurrent Giant Cell Tumour of Distal End Radius: Treatment and Outcomes After Further Surgeries

**DOI:** 10.7759/cureus.27451

**Published:** 2022-07-29

**Authors:** Umesh Yadav, Mohit Singla, Ajay Sheoran, Kshitij Behera, Abhishek Garg, Zile Singh Kundu, Anand Gupta, Ashish Devgun, Ravi Kumar, Puneet Yadav

**Affiliations:** 1 Department of Orthopaedics, Pandit Bhagwat Dayal Sharma Post Graduate Institute of Medical Sciences, Rohtak, IND; 2 Department of Surgical Oncology, Homi Bhabha Cancer Hospital, Varanasi, IND; 3 Department of Surgical Oncology, Positron Multi Speciality & Cancer Hospital, Rohtak, IND

**Keywords:** bone tumors, distal radius gct, wrist arthrodesis, resection, extended curettage, recurrence

## Abstract

Introduction: Distal end radius is the second most common location for giant cell tumours (GCTs) followed by the knee. Like at any other location, they are treated with extended curettage or resection but reportedly have an increased propensity for recurrence. This study aims to treat the recurrent distal end radius GCTs and their outcome after further surgeries.

Patients and methods: This study was conducted retrospectively from 2009 to 2021 and included 32 patients with recurrent distal end radius GCTs with a mean age of 29.53 years (range: 18-45 years). Twenty-five recurrences occurred after curettage and seven after resection. Twelve lesions were treated with further extended curettage. Nineteen recurrent lesions were treated with resection and arthrodesis. One out of two soft tissue recurrences was treated with en bloc resection. The mean follow-up period was 45.25 months (range: 24-120).

Results: The patients with joint preservations treated with further curettage and those where resection of soft tissue recurrences was done with salvage of joint had better functional outcomes with a mean Musculoskeletal Tumor Society (MSTS) score of 26.53 (Range: 22-30). The cases with arthrodesis had an average score of 23.75 (Range: 20-26). The overall average MSTS score was 24.89.

Conclusions: We conclude that local recurrence contained within the bone can be re-curetted. The isolated soft tissue recurrences can be re-excised. The bony lesions with extensive soft tissue extension should be treated with resection and reconstruction. The re-recurrence rate after further adequate treatment does not increase much.

## Introduction

Giant cell tumours (GCTs) represent about 5% of all the primary bone tumours and 20% of benign primary bone tumours with the peak incidence between 20-40 years and slight female predominance [1]. Campanacci et al. radiologically graded this tumour in three grades depending upon the destruction of the bone and its extension into the soft tissue [2]. Although this tumour has been studied extensively, the ideal treatment is yet to be achieved [3]. The local recurrence after simple curettage has been more than 50%. Extended curettage using liquid nitrogen, chemicals cauterization with phenol and alcohol, high-speed burring, pulsatile lavage, and thermo-coagulation followed by packing of the resultant cavity with polymethylmethacrylate (PMMA), bone grafts, and bone graft substitute is now the treatment option for grade 1 and 2 GCTs in long bones [3-6]. Local recurrence rates after such treatment have been reported from 0% to 25% [4-5,7]. Radical surgery like en bloc resection is advocated to avoid local recurrence [2,5-7]. However, this increases the morbidity because of the juxta-articular location of this tumour requiring arthrodesis. The grade 3 lesions with extension in the soft tissues or into the joint and in cases with less than 2/3rd circumferential cortex of the bone intact, which are not amenable to extended curettage have to be treated by resection and suitable reconstruction. The local recurrence after such treatment is about 5%. What to do and how to treat the local recurrences of distal end radius GCTs has been scarcely discussed in the literature, with opinions ranging from further intra-lesional curettage to resections [7,8]. We are reporting our experience of managing 32 patients with recurrent distal end radius GCTs.

## Materials and methods

This retrospective study was conducted at a tertiary level health institute, Pandit Bhagwat Dayal Sharma Post Graduate Institute of Medical Sciences, Rohtak, India. It included 32 patients (20 females and 12 males) with recurrent distal end radius GCTs between 2009 and 2022, with a mean age of 29.53 years (range: 18-45 years). The records of the patients were retrieved from the Orthopaedic Oncology clinic and the Department of Orthopaedics. The plain x-rays in two views were studied in all the cases. Proper staging using MRI or CT scan of the local site along with x-ray chest was done. The x-rays were evaluated as per Campanacci et al. radiological grading [2] and compartmental extension using Enneking et al. staging systems [9-11]. The radiographs were reviewed and studied by the musculoskeletal radiologist in collaboration with the operating surgeon. The biopsy confirmed the diagnosis and ruled out any malignant change. Thereafter the definitive surgery was planned. All the recurrent lesions were benign GCTs and none showed the malignant change in this series. All the cases were evaluated histopathologically by a pathologist trained in musculoskeletal tumour pathology.

Surgical technique

Extended curettage and re-filling of the cavity with bone grafts were carried out in grade 1 and 2 recurrent lesions (n=12). In these cases, the site of recurrence was ascertained and defined preoperatively by MRI. All the previous grafts from the site were removed after making a liberal window. The standard extended curettage was performed using sharp curettes, high-speed burrs, electro-coagulation, and pulsatile lavage. We performed only mechanical curettage and did not use phenol, alcohol, or liquid nitrogen. A total of 18 patients (56.25%) presented with Grade 3 lesions as per Campannaci staging, out of which 16 patients presenting with tumour extension into the soft tissues with little remaining bone precluding extended curettage were treated with en bloc resection and reconstruction. Recurrent GCT of distal end radius in a 22-year-old female treated with resection and wrist arthrodesis has been shown in Figure 1. The dissection of all important neurovascular and salvageable musculotendinous structures was performed for the preservation of functions. The tissue plains were not clearly demarcated due to the scar of previous surgery. Two patients (6.25%) presented with isolated soft tissue recurrences without any bony involvement. Both patients underwent en-block excision with a satisfactory functional outcome.

**Figure 1:** Recurrent GCT of distal end radius in a 22-year-old female treated with resection and wrist arthrodesis. (A) Preoperative radiograph showing recurrent GCT in distal end radius; (B) Intra-operative picture; (C) Postoperative radiograph showing resection and wrist arthrodesis; (D) Histological picture of patient with recurrent GCT (H&E stain); (E) and (F) showing functional outcome GCT: giant cell tumour; H&E: Hematoxylin and eosin

Follow-up

The sutures were removed after two weeks. The patients were followed up monthly for three months, three-monthly for the next two years, six-monthly for the next five years, and thereafter yearly. The mean follow-up period was 36.97 months (range 23- 120 months). The plain x-rays of the local site and chest were done at three months, six months, one year, and thereafter annually.

## Results

The details of the patients and grading (Campanacci) of tumours are depicted in Table 1.

**Table 1:** Descriptive patient demographics data

Variable	Number	Percent
Gender		
Male	12	37.5
Female	20	62.5
Grade (Campanacci)		
Grade-I	2	6.25
Grade-II	10	31.25
Grade-III	20	62.5

There were 20 female and 12 male patients. The mean age was 29.53 years (range: 18-45 years). Sixteen recurrences were noticed within six months of the first surgery, 10 within one year, and six presented at 18 months after surgery. There were 25 recurrences after curettages and seven after resections. Twenty-six patients with recurrences were treated initially outside by non-oncological orthopaedic surgeons. Thirty-two recurrences were either contained within the bone or with extension into the soft tissues and two isolated recurrences in soft tissues. These osseous recurrent lesions were graded as per Campanacci et al. radiologic grading as grade 1 (n=2, contained within the bone with no cortical expansion), grade 2 (n=10, lesions with expansion of the cortex), and grade 3 (n=18, lesions with extension into the soft tissues). The remaining two were soft tissue recurrences and were taken as grade 3. A female patient aged 30 years with soft tissue recurrence, which was treated with en bloc resection of the tumour, has been shown in Figure 2.

**Figure 2:** Soft tissue recurrence in a 30-year-old female. (A) Preoperative radiograph showing soft tissue recurrence; (B) and (C) Intra-operative picture; (D) Resected specimen; (E) Histological picture of patient with recurrent GCT (H&E stain); (F) Postoperative radiographs showing en bloc resection GCT: giant cell tumour; H&E: Hematoxylin and eosin

Re-extended curettage was done in 12 cases and the resultant cavities were filled with autologous bone grafts in three and with PMMA cement in the other nine cases. A total of 19 cases required resection of recurrence and reconstruction with arthrodesis). A fibular autograft was used for the arthrodesis in nine patients while ulna was transposed in 10 cases. Recurrent GCT of distal end radius in a 20-year-old female who was treated with resection and wrist arthrodesis with centralization of ulna has been shown in Figure 3.

**Figure 3:** Recurrent GCT of distal end radius in a 20-year-old female. (A) Preoperative radiographs showing recurrent GCT of distal end radius; (B) Postoperative radiograph showing resection and wrist arthrodesis with centralization of ulna; (C), (D), (E) Intra-operative pictures GCT: giant cell tumour

Two soft tissue recurrences after previous resections were treated with en bloc resection. Out of these two, one patient where after resection of lower end radius with no reconstruction was done by previous treating surgeon we performed arthrodesis of the wrist with centralization of the ulna. Table 2 illustrates the various treatment modalities used.

**Table 2:** Treatment data and complication

Variable	Number	Percent
Treatment		
Extended Curettage	12	37.5
Extended Curettage + Bone Grafting	3	9.37
Extended Curettage + Bone Cement	9	28.13
Resection & arthrodesis	19	59.3
En bloc resection of soft tissue	1	3.12
Complication		
Non-union at graft host bone junction	1	3.12
Infection	1	3.12
Rerecurrence	1	3.12
Implant related pain	1	3.12

Oncological results

One patient with recurrent GCT of distal radius developed pulmonary metastasis on subsequent follow-up. However, the patient was lost on sequential follow-up. Histopathologically, there was no case of malignant transformation or malignant GCT as such in this series.

Functional results

The functional status was assessed using the MSTS scoring system and Table 3 depicts the data regarding the same. The patients with joint preservations where further curettage was performed; those where resection of soft tissue recurrences was done with salvage of joint (n=13) had good functional outcomes with a mean MSTS score of 26.53 (Range: 22-30). The cases with arthrodesis (n=19) had an average MSTS score of 23.75 (Range: 20-26). Overall MSTS score of our series of 32 patients was 24.89 (Range: 20-30).

**Table 3:** Functional result according to MSTS score MSTS: Musculoskeletal Tumor Society

Type of Surgery	Number	Percentage	Mean	Range
Joint preservation surgery	13	40.6	26.53	22-30
Wide resection & arthrodesis	19	59.4	23.75	20-26
Overall	32	100	24.89	20-30

Complications

There was a superficial infection in one case, which was managed with intravenous antibiotics. . One patient experienced implant-related pain, which was managed by removing the prominent Kirschner wire. In one patient, non-union at the graft-host bone junction was observed, which was treated by autogenous bone grafting.

## Discussion

The clinical and biological behaviour of GCTs ranges from slow-growing latent lesions to active and locally aggressive tumours with a tendency for local recurrence [1-7]. Depending on the kind of treatment and the local extent of the lesion, the recurrence rates have been reported between 0% to 65% [7,12-16]. There have been ongoing efforts to reduce the recurrence, which with extended curettage along with adjuvants has been brought down to less than 25%. With wide resection, it has been brought down to about 5% but with added morbidity [17]. Disease clearance remains the primary aim and preservation of function is secondary.

The location/site of recurrence in the GCT is either on the surface of the bone in the cavity after curettage or in the soft tissues due to seedling or microscopic disease left behind after excision. When recurrence occurs after the curettage, this appears as lysis between the filler (bone graft/bone substitute or cement) and the host bone in x-rays. Such recurrences are better appreciated and can be picked up early in the cementation as there appears larger rim of lysis between homogenous cement and host bone as compared to cavities filled with bone grafts or bone substitutes, which are not as homogenous as cement [18]. During resection, if there is spillage due to capsule burst, there is seedling and recurrence in the soft tissues. To lessen the recurrence, curettage needs to be thorough and exhaustive using sharp curettes, high-speed burr, electro-coagulation, and pulsatile lavage. It is pertinent to mention here that function should not come at the price of unacceptably high re-recurrence rates.

When intralesional curettage is performed, local adjuvants such as PMMA, phenol, cryotherapy, and hydrogen peroxide have been reported to reduce the risk of local recurrence [7,13,17,19-20]. The treatment outcomes of the local recurrences and the incidence of re-recurrence have been barely discussed in the literature [3,7,21]. Table 4 shows the literature review in cases of GCT recurrence.

**Table 4:** Literature review of cases of GCT recurrence GCT: giant cell tumor; PMMA: polymethylmethacrylate

Study	Number of cases of recurrent GCTs	Treatment modality used	Recurrence rate
Turcotte et al., 2002 [16]	28	Intralesional curettage	35%
von Steyern et al., 2006 [3]	19	Curettage and PMMA filling	14%
Balke et al., 2009 [13]	66	High speed burring + PMMA	21.75%
		Intralesional curettage without any additive therapy	58.8%
Klenke et al., 2011 [7]	46	Wide resection	6%
		Intralesional curettage	32%
		Intralesional curettage +PMMA	14%
		Intralesional curettage +bone grafting	50%
Cheng et al., 2015 [22]	15	Curettage and blurring	18.75%

The use of PMMA instead of bone grafting as filler is associated with a decreased risk of tumour recurrence [7]. Balke et al. in a series of 66 patients with recurrent GCTs of the axial skeleton and the extremities observed that high-speed burring plus along with the use of PMMA decreased the recurrence rate as compared to the intralesional curettage without any additive therapy [21]. Cheng et al. studied 15 cases of recurrent GCT out of which 14 patients were treated with curettage and burring [22]. von Steyern et al. studied 19 patients with recurrent GCTs out of which 14 were treated with repeat curettage and PMMA filling with good to excellent outcomes [3]. PMMA reduces recurrence due to its thermal and toxic effects on tumour cells [23-24]. Further, when PMMA is used, the surgeon has a more aggressive approach to tumour removal leading to a big cavity, and the better mechanical property of cement reduces the risk of collapse of the cavity. Thus, the thorough tumour removal along with heat-mediated tumour cell death has an additive effect on the reduction of recurrence [17,23-24].

Wide resection lowers the recurrence rate as compared to the patients treated with intralesional curettage [12,15,19-20,25] but it requires complex reconstructions associated with greater functional impairment [7]. Twelve patients qualified for further extended curettage as per their extent of the disease and had one recurrence (3.12%). Two soft tissue lesions were simply resected en bloc with no recurrence. Thus, there was one recurrence (3.12%). This is comparable with the literature [7,21].

As per our experience, we hereby present treatment guidelines for patients with GCT recurrence in Figure 4. For intra-lesional surgery, we also observed that the quality of the mechanical curettage is most important. The use of a high-speed burr and filling the cavity with PMMA reduces re-recurrence [7,21,23-25]. After recurrence the tissue plains are not as clear; so one has to be meticulous in the dissection of important neurovascular structures, particularly in the cases previously treated with resection. But all the lesions could be well managed with a particular treatment, i.e., extended curettage by filling the cavity with cement or bone grafts, or resection and reconstruction with respect to the grade of the lesion just like primary lesions in the same grade and stage. After the second surgery, the functional results did not deteriorate much. The histopathology of these lesions after recurrence and re-recurrence revealed that all the lesions remained benign with no change in biological behaviour in this series.

**Figure 4:** Treatment guidelines for patients with GCT recurrence Image credits: Ajay Sheoran GCT: giant cell tumour

The risk of pulmonary metastases in patients with GCT is 2-10%. Only one patient in our study had pulmonary metastases (3.12%). Such pulmonary lesions are usually accompanied by local recurrence but are not fatal. Every patient with a local recurrence of GCT should be examined with a CT scan of the chest. Once recurrence is confirmed, treatment includes wedge resection, radiotherapy, and chemotherapy.

Another factor having a significant impact on recurrence rate is the primary management of these cases by general orthopaedic surgeons not specifically trained in orthopaedic oncology. In our study, twenty-six patients were referred by general orthopaedic surgeons. So we suggest that the recurrences should be treated meticulously, followed up vigilantly, and preferably by an oncologically trained orthopaedic surgeon. If these are further curetted adequately or excised properly as per the extent of the lesion, chances of re-recurrence do not increase in skilled hands. However, further treatment with the curettage or excision becomes difficult due to scarring and fudging of tissue planes compared to the primary de novo lesions and should be treated by a person with expertise in this field. The strength of this study is that all the cases were treated in one institution by a single orthopaedic oncological surgeon and his team. There is a good length of follow-up of 2-10 years in a reasonably large series of 32 patients. All the cases were evaluated histopathologically by the pathologists trained in musculoskeletal onco-pathology and the images by the experienced radiologist in collaboration with the operating surgeon. The limitations of this study include that 26 patients were treated elsewhere by general orthopaedic surgeons initially and then referred to us after recurrence. It is difficult to be certain in how many of these cases it was really a microscopic disease or was a residual macroscopic tumour. The quality of curettage performed by them is not ascertained. There is no similarity of the cases in view of the previous treatment as we have included the cases of recurrence after curettage as well as after resection.

## Conclusions

We conclude that local recurrence of GCT after curettage in long bones if contained within the bone and not extending into the soft tissue, can be successfully treated with further curettage and cementing and/or bone grafts with minimal risk of increased morbidity. More extensive surgery in an attempt to obtain wide margins is not required as it increases morbidity with no significant gain with respect to the cure of the disease. The soft tissue local recurrences can be re-excised. The grade 3 lesions with extensive soft tissue extension should be treated with resection and reconstruction exactly in a similar fashion as the primary lesions of the same grade. The re-recurrence rate after further proper treatment does not increase much. These lesions should preferably be treated by orthopaedic surgeons with adequate training in this field.
